# Glycolysis promotes caspase-3 activation in lipid rafts in T cells

**DOI:** 10.1038/s41419-017-0099-z

**Published:** 2018-01-19

**Authors:** Michael A. Secinaro, Karen A. Fortner, Oliver Dienz, Angela Logan, Michael P. Murphy, Vikas Anathy, Jonathan E. Boyson, Ralph C. Budd

**Affiliations:** 1 Vermont Center for Immunology and Infectious Diseases, Larner College of Medicine, University of Vermont, Burlington, VT USA; 2 Department of Surgery, Larner College of Medicine, University of Vermont, Burlington, VT USA; 3 MRC Mitochondrial Biology Unit, University of Cambridge, Cambridge, UK; 4 Department of Pathology and Laboratory Medicine, Larner College of Medicine, University of Vermont, Burlington, VT USA

## Abstract

Resting T cells undergo a rapid metabolic shift to glycolysis upon activation in the presence of interleukin (IL)-2, in contrast to oxidative mitochondrial respiration with IL-15. Paralleling these different metabolic states are striking differences in susceptibility to restimulation-induced cell death (RICD); glycolytic effector T cells are highly sensitive to RICD, whereas non-glycolytic T cells are resistant. It is unclear whether the metabolic state of a T cell is linked to its susceptibility to RICD. Our findings reveal that IL-2-driven glycolysis promotes caspase-3 activity and increases sensitivity to RICD. Neither caspase-7, caspase-8, nor caspase-9 activity is affected by these metabolic differences. Inhibition of glycolysis with 2-deoxyglucose reduces caspase-3 activity as well as sensitivity to RICD. By contrast, IL-15-driven oxidative phosphorylation actively inhibits caspase-3 activity through its glutathionylation. We further observe active caspase-3 in the lipid rafts of glycolytic but not non-glycolytic T cells, suggesting a proximity-induced model of self-activation. Finally, we observe that effector T cells during influenza infection manifest higher levels of active caspase-3 than naive T cells. Collectively, our findings demonstrate that glycolysis drives caspase-3 activity and susceptibility to cell death in effector T cells independently of upstream caspases. Linking metabolism, caspase-3 activity, and cell death provides an intrinsic mechanism for T cells to limit the duration of effector function.

## Introduction

The balance of cell proliferation and cell death is critical for the maintenance of stable cell numbers and tissue homeostasis. Thus, it is perhaps not surprising that these opposing processes may be mechanistically linked in various cell types, including cancer^1,2^. During an immune response, T lymphocytes undergo a period of very rapid proliferation. During this expansion, T cells also become susceptible to T-cell receptor (TCR) restimulation-induced cell death (RICD)^3,4^. However, the link between proliferation and susceptibility to death remains poorly understood^5^.

Changes in cellular metabolism are well recognized to play a critical role during an effective immune response. Resting naive T lymphocytes, upon activation, undergo a dramatic metabolic shift from oxidative phosphorylation to aerobic glycolysis^6–8^. The switch to a largely glycolytic state allows the cell to generate the synthetic capacity needed for rapid proliferation and effector function, such as cytokine production. In a similar manner, B cells and dendritic cells also utilize glycolysis upon activation to enable their effector functions^9,10^. Recent studies have further indicated that the metabolic state of effector T cells helps determine their subset differentiation^11^. Differing metabolic states are also known to be involved in the specification of T-cell memory, with central memory T cells exhibiting high oxidative phosphorylation and effector memory T cells being more glycolytic^12–14^.

It is well appreciated that cell death and metabolism are closely linked. Glycolytic enzymes can be induced by the same transcription factors that upregulate the expression of anti-apoptotic proteins such as BCL-xL^15^. Other proteins with metabolic function, such as cytochrome c, are directly involved in cell death^15,16^. When released from the mitochondria, cytochrome c activates caspase-9, which then cleaves caspase-3 and induces apoptosis. Caspase-3 can be alternatively activated through cleavage by caspase-8, which is activated by death receptors such as Fas (CD95). However, little is known regarding possible links between metabolism and caspase activity.

Although caspases were originally defined for their role in cell death, it is now appreciated that caspases perform many functions in cells in addition to cell death^17,18^. This is particularly well established for caspase-8, an initiator caspase that can induce apoptosis upon ligation of a death receptor^19^, but can also allow cell proliferation by inhibiting formation of the necroptosome and induction of necroptosis^20^. Active caspase-3, a critical downstream mediator of apoptosis, has also been observed in non-dying cells and is implicated in skeletal muscle differentiation^21^, T-cell anergy^22^, B-cell cycling^10^, and erythrocyte maturation^17^. However, these studies did not examine how caspase-3 activity is being regulated in these non-apoptotic situations. Moreover, an explanation has been lacking for the molecular switch between TCR-stimulated proliferation of naive T cells vs. induction of cell death in effector T cells^3,4^.

Given the involvement of caspases in both cell death and non-death functions, regulation of caspase activity and its location in cells are of paramount importance in determining cell fate. We have observed that T cells grown in interleukin (IL)−2 vs. IL-15 have similar amounts of total pro-caspase-3, but IL-2-cultured T cells have a substantially higher level of active caspase-3, and as a result are much more susceptible to RICD^23^. IL-15-cultured T cells are resistant to this form of cell death, in part due to the high levels of reactive oxygen and nitrogen species that lead to the redox modification of a critical cysteine in the active site of caspase-3, resulting in its inactivation^23–25^. IL-2 and IL-15 also induce very different metabolic states in T cells; IL-2 promotes glycolysis, whereas IL-15 upregulates oxidative phosphorylation^12^. We now observe that caspase-3 activity in non-dying effector T cells is largely a function of their glycolytic state. Inhibition of glycolysis by a variety of methods reduces caspase-3 activity and protects T cells from RICD. In addition, IL-15-cultured T cells further reduce caspase-3 activity through its inactivation by glutathionylation. These findings underscore the importance of cellular metabolism in the regulation of caspase-3 activity and susceptibility toward cell death.

## Results

### IL-15 induces mitochondrial ROS and glutathionylation of caspase-3

To investigate the influence of cell metabolism on caspase activity, we initially modeled two metabolic states in vitro using cytokines that are known to promote very different levels of glycolysis following T-cell activation: IL-2, which upregulates glycolysis, and IL-15, known to induce a non-glycolytic state of mitochondrial respiration^12^. To mimic an immune response in vitro, purified naive T cells were activated with anti-CD3/CD28 in the presence of IL-2 for 2 days, and then removed from stimulation and propagated in IL-2 for an additional day. The activated T cells were then washed thoroughly to remove exogenous cytokines and recultured in medium containing either IL-2 or IL-15 for an additional 3 days. In agreement with previous observations^12^, IL-15-cultured T cells manifested high mitochondrial respiration, as reflected by a high oxygen consumption rate (OCR; Fig. 1a). Consistent with these findings, complex I activity of the electron transport chain was higher in IL-15-cultured T cells than in IL-2-cultured T cells (Figs. 1b, c). Complex I is known to generate reactive oxygen species (ROS)^26^, and we determined that IL-15 induced a greater amount of mitochondrial ROS compared to IL-2 (Fig. 1d) as measured using the mitochondria-targeted probe mitoboronic acid (MitoB)^27^. MitoB is converted to mitophenol (MitoP) upon reaction with mitochondrial hydrogen peroxide, and the levels of MitoB and MitoP are then measured by liquid chromatography tandem mass spectrometry and expressed as a ratio of MitoP to MitoB^27^.

**Fig. 1:** IL-15 drives increased oxygen consumption, complex I activity, and mitochondrial ROS Anti-CD3/CD28-activated T cells were cultured for 3 days in IL-2 or IL-15. **a** Oxygen consumption rate (OCR) was measured by extracellular flux analysis. *O* Oligomycin A (inhibitor of ATP synthase), *F* FCCP (uncoupler of the electron transport chain), *R/A* Rotenone and Antimycin (inhibitors of complexes I and III, respectively; mean ± S.D. of four replicates within the one experiment shown. The graph is representative of two independent experiments). **b** Complex I activity was measured in mitochondrial (Mito) and cytosolic (Cyto) fractions of IL-2- or IL-15-cultured T cells (the graph is representative of two independent experiments). **c** Complex I rates of activity in (**b**) for mitochondrial fractions, normalized to the rate of activity of complex I in mouse liver mitochondria (unpaired *t*-test; *p < 0.05; mean ± S.D. of data from two independent experiments). **d** Mitochondrial ROS were measured by the conversion of mitoboronic acid (MitoB) to mitophenol (MitoP), and the ratio of MitoP/MitoB was measured by liquid chromatography tandem mass spectrometry (paired *t*-test; *p < 0.05; mean ± S.E.M. of means from three independent experiments)

ROS can promote protein glutathionylation, a process that results in the reversible modification of a cysteine by glutathione^28^. Caspase-3 has been shown previously to be inactivated in HL-60 cells by the glutathionylation of the critical cysteine in the enzymatic pocket^25^. We therefore investigated the possibility that caspase-3 is glutathionylated in IL-15-cultured T cells. Glutathionylated proteins were immunoprecipitated and immunoblotted for caspase-3 (Fig. 2a). Caspase-3 was glutathionylated to a considerably greater extent in the IL-15-cultured T cells compared to IL-2 (Fig. 2b). Of interest, the glutathionylation was observed specifically on cleaved caspase-3 (Fig. 2a). This implies that full-length pro-caspase-3 was initially cleaved and then inactivated by glutathionylation.

**Fig. 2:** IL-15 induces glutathionylation of caspase-3 Anti-CD3/CD28-activated T cells were cultured in IL-2 or IL-15 for 3 days before lysis. **a** Glutathione immunoprecipitation (GSH IP) was performed on whole-cell lysates (WCL). Immunoprecipitations were conducted alongside a reduced control (+DTT) and an IgG control (IgG). The WCL and GSH IP were immunoblotted for caspase-3 (the immunoblot is representative of three independent experiments). **b** Densitometry of cleaved caspase-3 detected in the IL-2 and IL-15 GSH IP lanes in (**a**), indicative of glutathionylated cleaved caspase-3 (paired *t*-test; *p < 0.01; mean ± S.D.; *n* = 3 independent experiments). **c** ROS were measured by flow cytometry using DCFDA in IL-2- or IL-15-cultured T cells in the presence or absence of 200 nM mitoquinone (MitoQ) for 4 h (two-way ANOVA with Sidak’s correction; data indicate a fold change compared to IL-2 DMSO control; *NS *not significant; *p < 0.05; mean ± S.E.M.; *n* = 3 independent experiments). **d** Caspase activity was measured by DEVD rhodamine fluorescence in IL-2- or IL-15-cultured T cells with or without MitoQ (two-way ANOVA with Sidak’s correction; *NS *not significant; *p < 0.05; mean ± S.D. of three replicates within the one experiment shown. The graph is representative of two independent experiments). **e** IL-2- or IL-15-cultured T cells were incubated with MitoQ (200 nM) or DMSO for 24 h. Restimulation-induced cell death was then promoted by 16 h anti-CD3 restimulation followed by Live/Dead staining and flow cytometry (two-way ANOVA with Tukey’s correction; *NS *not significant; mean ± S.D. of two replicates)

Given that IL-15 induced a greater amount of mitochondrial ROS compared to IL-2 (Fig. 1d), we examined the effect of quenching mitochondrial ROS on overall caspase activity in activated T cells. IL-2- and IL-15-cultured T cells were incubated with the mitochondria-targeted antioxidant mitoquinone (MitoQ) to quench mitochondrial ROS^29^. MitoQ treatment of IL-15-cultured T cells, but not IL-2-cultured T cells, induced a reduction in ROS (Fig. 2c). The lack of effect of MitoQ in IL-2-cultured T cells may reflect a non-mitochondrial source of ROS, such as cytoplasmic NADPH oxidases. Consistent with these findings, MitoQ did not alter caspase activity in IL-2-cultured T cells, but did slightly increase caspase activity in IL-15-cultured T cells, although not to the level of caspase activity in IL-2-cultured T cells (Fig. 2d). Consistent with these findings, treatment with MitoQ did not affect the sensitivity of IL-2- or IL-15-cultured T cells to death, either before or after restimulation (Fig. 2e). Thus, mitochondrially derived ROS partially contributed to the low level of caspase activity in IL-15-cultured T cells, but were not solely responsible for the decreased sensitivity to RICD. We therefore considered that the pronounced metabolic shift to glycolysis during T-cell activation might also influence the activity of certain caspases and sensitivity to RICD.

### Glycolysis drives caspase-3 activation

Glycolysis was measured by extracellular acidification rate (ECAR) in naive T cells, effector T cells (day 6 after activation), and late effector T cells (day 10 after activation). Glycolysis increased initially from naive to day 6 T cells, and then decreased from day 6 to day 10 (Fig. 3a). These changes were greater in the IL-2-cultured T cells than IL-15. IL-2 signaling is known to drive glycolysis^12^, and the kinetics of glycolysis in T cells grown in IL-2 closely paralleled the levels of surface IL-2 receptor α (CD25) expression, which also peaked and declined over a nearly identical timespan (Fig. 3b). These results are consistent with previously reported kinetics of CD25 expression^30^. Concomitant with the rise of glycolysis and surface CD25 expression following T-cell activation, we observed an increase in total caspase activity. T cells propagated in IL-2 continued to increase caspase activity until a peak on day 6, after which it declined through day 10, closely paralleling ECAR and CD25 expression (Fig. 3c). As a result of the culturing system and the introduction of IL-15 on day 3, the first measurements of caspase activity and CD25 expression occurred on day 4 for IL-15-cultured T cells. In the presence of IL-15, CD25 expression and caspase activity remained at a consistently low level throughout the same 10-day period (Fig. 3c). The largest difference in caspase activity between IL-2- and IL-15-cultured T cells was on day 6. We also measured the level of active caspase-3 by flow cytometry, and found it to be greater in IL-2-cultured T cells compared with IL-15-cultured T cells on day 6 (Fig. 3d). Whereas caspase-3 activity was detected in live IL-2-cultured T cells, activity was much higher in cells in which death was induced through Fas stimulation (Fig. 3d). Thus, the intermediate levels of active caspase-3 in proliferating T cells were not due to contaminating dead cells, but rather were present in all IL-2-cultured T cells.

**Fig. 3:** Caspase activity parallels glycolysis and CD25 expression in T cells **a–c** T cells were activated with anti-CD3/CD28 for 2 days and cultured in IL-2 for a third day. T cells were then washed and cultured in IL-2 or IL-15 for an additional 7 days. **a** Baseline extracellular acidification rate (ECAR) was measured by extracellular flux analysis on days 0, 6, and 10 (two-way ANOVA with Tukey’s correction; *NS *not significant; *p < 0.01; mean ± S.E.M. of means from three independent experiments). **b** CD25 expression measured daily by flow cytometry (the graph is representative of two independent experiments). **c** Caspase activity was measured daily by DEVD rhodamine release (mean ± S.D. of three replicates within the one experiment shown. The graph is representative of two independent experiments). **d** Anti-CD3/CD28-activated T cells were cultured in IL-2 or IL-15 for 3 days. For a positive control, IL-2-cultured T cells were incubated with FasL for 1.5 h to induce caspase-3 activity and cell death. Cells were stained for intracellular active caspase-3 and analyzed by flow cytometry (the graph is representative of three independent experiments). **e**,** f** Purified CD4^+^ T cells were differentiated into Th1, Th2, and Treg subsets by activation with anti-CD3/CD28 for 2 or 3 days along with the appropriate cytokines (see Materials and Methods). T-cell subsets were then cultured for an additional 2 or 3 days in IL-2 according to an established protocol^11^. **e** Baseline ECAR was measured by extracellular flux analysis (one-way ANOVA with Tukey’s correction; **p < 0.0001; mean ± S.D. of five replicates within the one experiment shown. The graph is representative of two independent experiments). **f** Caspase activity was measured by DEVD rhodamine fluorescence (one-way ANOVA; **p < 0.0001; mean ± S.D. of three replicates within one experiment. The graph is representative of two independent experiments)

To extend the observed correlation of glycolysis with caspase activity, we examined CD4^+^ T-cell functional subsets, which have been shown to have varying levels of glycolytic activity^11^. In vitro-differentiated T helper (Th)1 and Th2 cells were reported to have high levels of glycolysis, being slightly higher in Th2 cells. By contrast, in vitro-differentiated T regulatory (Treg) cells had low levels of glycolysis. Purified naive CD4^+^ T cells were differentiated into Th1, Th2, and Treg cells in vitro and their caspase activity was measured. Caspase activity was highest in the Th2 subset and lowest in the Treg subset, matching glycolytic activity (Figs. 3e and f).

These collective findings suggested that glycolysis and caspase activity might be causally linked. We thus examined more directly the effect of glycolysis on caspase activity. To inhibit glycolysis, IL-2-cultured T cells were incubated with 2-deoxy-D-glucose (2-DG), a glucose analog that blocks glucose catabolism after phosphorylation by hexokinase^31^. As an inhibitor of glycolysis, 2-DG could potentially induce cell death in highly glycolytic IL-2-cultured T cells. To reduce contamination by dead cells, the 2-DG cell cultures were centrifuged over Histopaque. The inhibition of glycolysis by 2-DG was confirmed by measuring a decrease in ECAR (Fig. 4a). In parallel, caspase activity was also decreased, in a dose-dependent manner, in IL-2-cultured T cells cultured with 2-DG (Fig. 4b). To confirm that the decrease in caspase activity was due to the inhibition of glycolysis and not an off-target effect of 2-DG, we also inhibited glycolysis by two other methods, culturing IL-2-cultured T cells with rapamycin or in a low-glucose medium. These treatments also reduced caspase activity in IL-2-cultured T cells (Fig. 4b) but not in IL-15-cultured T cells (Fig. 4c).

**Fig. 4:** Glycolysis regulates caspase activity in effector T cells Anti-CD3/CD28-activated T cells were cultured for 3 days in IL-2 with (**a**) 2-deoxyglucose (2-DG, 0–5 mM). Baseline ECAR was measured (one-way ANOVA with Dunnett’s correction; **p < 0.001; mean ± S.E.M. of means from three independent experiments). **b**,** c** Activated T cells were cultivated for 3 days in (**b**) IL-2 or (**c**) IL-15, in medium, 2-deoxyglucose (2-DG, 5 mM), without glucose (No glucose), Rapamycin (300 nM), or DMSO control. Caspase activity was measured by DEVD rhodamine fluorescence. Data indicate a fold change compared to the control (one-way ANOVA with Dunnett’s correction; *p < 0.05; **p < 0.001; mean ± S.D.; *n* = 3 independent experiments)

To determine whether the regulation of caspase activity by glycolysis was selective for certain caspases, we examined the levels of specific caspase activity in IL-2-cultured T cells in the presence or absence of 2-DG, using biotin-VAD (bVAD) to selectively precipitate only active caspases with streptavidin-coated Sepharose beads. Immunoblot analysis of the precipitates revealed that 2-DG caused a profound decrease in caspase-3 activity, but had no effect on the activities of the related effector caspase-7, nor the upstream caspase-8 or caspase-9 (Figs. 5a, b). The disparate levels of active caspase-3 in glycolytic vs. non-glycolytic T cells suggested that they might differ in their susceptibility to cell death following TCR restimulation. Day 6 IL-2-cultured T cells cultured with and without 2-DG were restimulated with anti-CD3. While 2-DG induced more cell death prior to restimulation (Fig. 5c), the 2-DG-treated cells were considerably more resistant to RICD (Fig. 5d). RICD is primarily mediated by Fas-ligand (FasL) signaling^32^. Therefore, we measured FasL by western blot and found expression to be highest in glycolytic IL-2-cultured T cells, and slightly less in non-glycolytic IL-15-cultured and 2-DG-treated T cells (Figs. 5e, f). However, the fact that the activities of caspases-8 and -9 were not affected by 2-DG suggests that FasL did not mediate caspase-3 activity in viable IL-2-cultured T cells.

**Fig. 5:** Activity of caspase-3, but not caspase-8 or caspase-9, is regulated by the glycolytic state of effector T cells Activated T cells were cultured for 3 days in IL-2 with or without 5 mM 2-DG. **a** Active caspases were selectively precipitated using biotin-VAD (bVAD) and streptavidin Sepharose beads, and immunoblotted for caspases-8, -9, -7, and -3 (the blot is representative of two independent experiments). **b** Densitometry of active caspase-8, -9, -7, and -3 in (**a**; for caspase-8, -9, and -3: two-way ANOVA with Sidak’s correction; for caspase-7: unpaired *t*-test; *NS *not significant; *p < 0.05; mean ± S.D. of two replicates). **c** Cell death was determined by Live/Dead staining after centrifugation over Histopaque (unpaired *t*-test; mean ± S.D.; **p < 0.01; *n* = 3 independent experiments). **d** Restimulation-induced cell death was promoted by 16 h anti-CD3 restimulation of IL-2-cultured T cells cultured with or without 2-DG, and cell death determined by Live/Dead staining using flow cytometry. Data indicate fold change compared to the unstimulated medium control (two-way ANOVA with Sidak’s correction; *NS *not significant; *p < 0.05; mean ± S.D. of two replicates; *n* = 2 independent experiments). **e** Cell lysates of T cells grown in the indicated conditions were immunoblotted for FasL. Controls included FasL-transfected 3T3 cells or mock-transfected 3T3 cells (the immunoblot is representative of two independent experiments). **f** Densitometry of FasL in (**e**; one-way ANOVA; *p < 0.05; **p < 0.01; mean ± S.D. of two replicates)

### Active caspase-3 is sequestered in membrane lipid rafts in effector T cells

Self-cleavage of caspases can occur when pro-caspases are clustered in close proximity^33^, such as in lipid rafts where caspase-8 is known to be active in effector T cells^34,35^. To determine whether caspase-3 was localized to membrane lipid rafts in effector T cells, lipid rafts were purified from both glycolytic, IL-2-cultured T cells, and non-glycolytic, IL-15-cultured T cells, and the resulting fractions were analyzed for caspase-3 cleavage and activity. In IL-2-cultured glycolytic T cells, pro-caspase-3 was present primarily in the non-raft fractions, and to a much lesser extent in the raft fractions (Fig. 6a, raft fractions: 3–5; non-raft fractions: 10 and 11). However, caspase-3 was extensively cleaved only in the lipid raft fractions. In the IL-15-cultured non-glycolytic T cells, pro-caspase-3 was also found predominantly in the non-raft fractions. Although caspase-3 was also observed to be cleaved primarily in the raft fractions of IL-15-cultured T cells, it was to a lesser extent than in IL-2-cultured T cells (Fig. 6b). Hence, the ratio of cleaved caspase-3 to pro-caspase-3 was greater in the lipid rafts of IL-2-cultured glycolytic T cells than in non-glycolytic IL-15-cultured T cells (Fig. 6c).

**Fig. 6:** IL-2-mediated glycolysis promotes the localization and cleavage of caspase-3 in lipid rafts Activated T cells were cultured for 3 days in IL-2 or IL-15. **a**,** b** Cells were sonicated before fractionation in an ultracentrifuge over an Optiprep density gradient. Fractions of 1 mL each were collected. A volume of 30 μL of each fraction was used to perform an immunoblot for capsase-3, GM-1 (lipid rafts), and paxillin (non-raft; the blot is representative of two independent experiments). **c** Densitometry of the ratio of cleaved capsase-3 to pro-caspase-3 in raft and non-raft fractions (*n* = 2 independent experiments). **d** bVAD precipitation of active caspases was performed on the indicated raft and non-raft fractions, and precipitates were immunoblotted for active caspase-3 (the blot is representative of two independent experiments). **e** Densitometry of active caspase-3 in raft and non-raft fractions (*n* = 2 independent experiments)

To confirm that the cleaved caspase-3 observed in lipid rafts was active, we performed a bVAD precipitation on the lipid raft fractions 3–5 and the non-raft fraction 11. Caspase-3 was found to be active at a much greater extent in the raft fractions of IL-2-cultured glycolytic T cells, compared with IL-15-cultured non-glycolytic T cells (Figs. 6d, e).

### Caspase-3 activity increases in effector T cells during influenza infection

To determine whether active caspase-3 is observed in activated T cells in vivo, mice were infected intranasally with influenza virus strain A/Puerto Rico/8/1934 H1N1 (Flu) and lymphocytes from the lung-draining mediastinal lymph node were analyzed after 6 days. Caspase-3 activity was measured in naive (CD44^low^) and proliferating effector (CD44^high^) CD4^+^ and CD8^+^ T cells (Fig. 7a). The percentage of active caspase-3-positive cells, as well as the median fluorescence intensity (MFI) of active caspase-3 staining, were increased in the CD44^high^ population of both CD4^+^ and CD8^+^ T cells after Flu infection, compared to the CD44^low^ population (Fig. 7b).

**Fig. 7:** Caspase-3 is active in vivo in proliferating T cells after influenza infection Mice received influenza virus strain A/Puerto Rico/8/1934 H1N1 virus (FLU) or PBS control intranasally and lymph nodes were extracted 6 days after infection. Mediastinal lymph node cells (flu-infected mice) or non-mediastinal lymph node cells (PBS control mice) were stained and analyzed by flow cytometry. **a** Representative contour plots of live CD4^+^ (left) or CD8^+^ (right) T cells from PBS control mice (top) or flu-infected mice (bottom) for CD44 vs. active caspase-3. The two rectangular inserts identify the CD44^high^ (upper) and CD44^low^ (lower) populations. All events to the right of the vertical line are positive for active caspase-3. Numbers represent the percentage of CD44^high^ or CD44^low^ gated cells that are positive for active caspase-3 (% + ), and the median fluorescent intensity of active caspase-3 (MFI). **b** Graphs of the percent positive cells for active caspase-3 (top) and MFI (bottom; two-way ANOVA with Tukey’s correction; mean ± S.D.; *p < 0.001, **p < 0.0001. *NS* not significant. *n* = 5 mice per group)

## Discussion

The present findings reveal that IL-2-mediated glycolysis increases caspase-3 activity and the consequential susceptibility of effector T cells to caspase-3-mediated cell death. IL-15, by contrast, drives low levels of glycolysis that favor low caspase-3 activity. The high amount of oxidative metabolism in IL-15-cultured T cells also promotes a further decrease in caspase-3 activity through its glutathionylation. Our data support a model by which glycolytic metabolism sets the stage for a high proliferative rate of effector T cells that is coupled to enhanced susceptibility to death cues through the activity of downstream effector caspase-3.

Cleavage of caspase-3 can be induced by upstream caspase-8 following Fas ligation, and by caspase-9 following cytochrome c release from the mitochondria. It is also possible for cleavage of caspase-3 to occur by self-activation when caspase-3 molecules are clustered in close proximity^33,36^. We observed that the levels of both caspase-8 and caspase-9 activity were similar between glycolytic and non-glycolytic T cells, suggesting that they are not likely to be the regulators of caspase-3 activity in these different metabolic states. The findings are also consistent with our previous observations that caspase-3 activity persists in effector T cells in which caspase-8 was deleted^37^. It is possible that translocation to the cell membrane, and particularly to lipid raft domains, allows the clustering of full-length inactive caspase-3, and could promote its proximity-induced autocleavage and activation^36,38^. Furthermore, while confined to lipid rafts, active caspase-3 may also be restricted in its access to substrates that might induce cell death.

Effector T cells and memory T cells have very different metabolic profiles. Similar to memory T cells derived in vivo, memory-like T cells can be generated in vitro through IL-15 signaling that promotes oxidative phosphorylation^12,13^. Consistent with those previous reports, we observed that compared to IL-2, IL-15-cultured T cells have elevated oxidative phosphorylation and mitochondrial ROS. Our findings further reveal that IL-15-cultured T cells manifest glutathionylation of caspase-3, which is known to inactivate caspase-3 at the critical cysteine in the enzymatic pocket^25^. Given that glutathionylation of caspase-3 was detected only of cleaved caspase-3 in IL-15-cultured T cells, this suggests that caspase-3 is being inactivated by glutathionylation after its cleavage. Along with our previous report of the inactivation of caspase-3 by S-nitrosylation^23^, these data show that in T cells caspase-3 can be inactivated by redox-dependent post-translational modifications, which are influenced by the metabolic state of the cell. Metabolically induced modifications of apoptotic caspases may be an important mechanism for memory T-cell formation.

The correlation between glycolysis and CD25 expression for in vitro-generated effector T cells is not surprising, given the known role of IL-2 in the induction of glycolysis in T cells. However, in vitro-differentiated Treg cells, despite expressing high levels of CD25, are not glycolytic, likely due to their derivation with TGFβ^11,39^. We observed that these cells have low caspase activity, indicating that caspase activity is a function of glycolysis rather than CD25 expression.

Proliferating T cells are known to be susceptible to cell death cues such as RICD^40,41^. Our data demonstrate independent increases in both FasL and caspase-3 activity in glycolytic IL-2-cultured T cells prior to TCR restimulation. Consistent with our observations, a study recently reported that human CD8^+^ T cells rapidly induced FasL protein following TCR restimulation only when glycolytic, rendering them more susceptible to RICD^42^. However, we do not feel that the caspase-3 activity or the caspase-8 activity in proliferating glycolytic T cells is due to Fas/FasL interactions for a few reasons. First, we observed no increased levels of active upstream caspase-8 in IL-2-cultured T cells despite more active caspase-3. Second, we have previously shown that Fas-deficient effector T cells express as much active caspase-8 as wild-type T cells^35^. Finally, reducing caspase-8 activity in effector T cells by deleting its regulator, c-FLIP, had no effect on the levels of active caspase-3^37^. Hence, the collective findings would indicate that the levels of active caspase-8 and caspase-3 in effector T cells are largely independent of one another as well as independent of Fas/FasL interactions.

At present, the full spectrum of function of caspase-3 activity in viable effector T cells is unclear. Other reports have noted a role for caspase-3 in T-cell anergy^22^, cleavage of p21 and cell cycling in B cells^10^, skeletal muscle differentiation^21^, and maturation of erythrocytes, macrophages, and dendritic cells^17^. The localization of active caspase-3 in membranes could provide access to substrates important to these functions, while simultaneously preventing the enzyme from cleaving pro-death substrates. While it is possible that the glycolytic state of cells may influence these other reported functions of caspase-3, the current findings nonetheless link metabolism to caspase-3 activity and thus provide a plausible regulatory mechanism of immune cell homeostasis.

## Materials and methods

### Mice

C57BL/6NJ male mice (Jackson Laboratory, Bar Harbor, ME) were housed in an Association for Assessment and Accreditation of Laboratory Animal Care International-approved facility at the University of Vermont Larner College of Medicine. Mice were used at 2–6 months of age, and protocols were approved by the Institutional Animal Care and Use Committee.

### Cell culture

T cells were purified from mouse lymph nodes (axillary, inguinal, brachial, and cervical) and spleens by negative selection as described previously^23^. Briefly, lymph nodes and spleens were homogenized through nylon mesh and red blood cells were lysed with Gey’s solution. Combined lymphocytes and splenocytes were incubated on ice for 30 min with the following antibodies: anti-CD11b (M1/70), anti-MHC class II (M5/114/15/2; a kind gift from M. Rincón, Larner College of Medicine, University of Vermont, Burlington, VT, USA), and anti-B220 (RA3-6B2). Cells were then rocked over magnetic goat anti-rat beads (Qiagen, Germantown, MD, USA) at a 10:1 bead:cell ratio for 45 min at 4 °C. Beads and bound cells were removed with a magnet. Naive T cells were cultured in RPMI-1640 (Corning, Manassas, VA, USA), supplemented with 25 mM HEPES, 100 U/mL penicillin–streptomycin (ThermoFisher Scientific, Waltham, MA, USA), 5% bovine calf serum (GE Healthcare HyClone, Logan, UT, USA), 2.5 mg/L glucose, 2 mM glutamine, 10 μg/mL folate, 1 mM pyruvate, and 50 μM 2-mercaptoethanol (RPMI-C) and stimulated on 10 μg/mL plate-bound anti-CD3 clone 145-2C11 (Bio X Cell, West Lebanon, NH, USA) and soluble anti-CD28 ascites clone 37–51 (1:1000), supplemented with 50 U/mL IL-2 (Cetus, Emeryville, CA, USA) at 37 °C, 5% CO_2_. After 2 days, activated T cells were removed from stimulation and cultured for an additional day in RPMI-C and 50 U/mL IL-2. Cells were then washed three times to remove cytokines and cultured for 2–3 more days in RPMI-C supplemented with either 50 U/mL IL-2 or 20 ng/mL IL-15 (a kind gift from Amgen, Thousand Oaks, CA, USA). For studies of the inhibition of glycolysis, T cells were activated for 2 days in RPMI-C medium supplemented with 50 U/mL IL-2. Cells were then washed three times and cultured in RPMI-C medium with 50 U/mL IL-2 and the indicated doses of 2-deoxy-D-glucose (Sigma-Aldrich, St. Louis, MO, USA) or rapamycin (MP Biomedicals, Solon, OH, USA) for 3 days, replacing media, cytokine, and inhibitor each day. IL-2-cultured T cells cultured in 2-deoxy-D-glucose were centrifuged over Histopaque-1077 (Sigma-Aldrich) to minimize the number of dead cells in the cultures prior to use in the assays. Alternatively, cells were washed and cultured with glucose-free RPMI-1640 (Corning) supplemented with 100 U/mL penicillin–streptomycin, 5% bovine calf serum, 2 mM glutamine, 10 μg/mL folate, 1 mM pyruvate, and 50 μM 2-mercaptoethanol (GF RPMI-C). Cells were then cultured in GF RPMI-C supplemented with the indicated decreasing concentrations of glucose for 3 days, replacing the media each day.

### Caspase activity assay

Caspase activity was measured using the Apo-ONE Homogeneous Caspase-3/7 Assay Kit (Promega, Madison, WI, USA) according to the manufacturer’s specifications. Samples were analyzed using a Synergy HT Plate Reader (BioTek, Winooski, VT, USA).

### Cell lysis and immunoblot analysis

Cells were lysed for 20 min on ice in Lysis Buffer A (0.5% Nonidet P-40, 150 mM NaCl, 20 mM Tris-HCl (pH 7.4), 10% glycerol, 2 mM sodium orthovanadate, and Complete Protease Inhibitor (Roche Diagnostics, Indianapolis, IN, USA)). Protein concentration was determined by Bradford Assay (Bio-Rad, Hercules, CA, USA). Lysates were boiled for 5 min in Laemmli loading buffer supplemented with 2-mercaptoethanol (2-ME). Proteins within the lysates were separated by SDS-PAGE on a 12% acrylamide gel and transferred to a polyvinylidene difluoride (PVDF) membrane (Bio-Rad). Membranes were blocked in 4% milk in Tris-buffered saline with 0.1% Tween-20 (American Bioanalytic, Natick, MA, USA) at room temperature for 1 h. The following antibodies were used for protein detection: anti-caspase-3, 585 rabbit polyclonal antibody (a kind gift from Dr. Yuri Lazebnik, Cold Spring Harbor Laboratories, Cold Spring Harbor, NY, USA), anti-caspase-8 (a kind gift from Dr. Andreas Strasser, The Walter and Eliza Hall Institute of Medical Research, Melbourne, Australia), anti-caspase-9, clone 5B4 (Stressgen Assay Designs, Ann Arbor, MI, USA), anti-flotillin (BD Biosciences), GM-1 HRP (Sigma-Aldrich), anti-paxillin, clone 165 (BD Biosciences), anti-FasL MAB5262 (R&D Systems, Minneapolis, MN, USA), anti-β-actin (Sigma-Aldrich), anti-mouse IgG HRP, anti-rabbit IgG HRP, and anti-rat IgG HRP (all from Jackson Laboratory). Densitometry was performed using Image Studio Lite v5 (LI-COR Biotechnology, Lincoln, NE, USA).

### bVAD active caspase precipitation

Cells were washed once with PBS containing 1% bovine serum albumin (PBS/1% BSA) and once with PBS, and then incubated on ice for at least 20 min with Lysis Buffer B (0.2% Nonidet P-40,150 mM NaCl, 20 mM Tris-HCl (pH 7.4), 10% glycerol, 2 mM sodium orthovanadate, and Complete Protease Inhibitor (Roche Diagnostics)) supplemented with 20 μM biotin-VAD-fmk (bVAD; MP Biomedicals). Protein was quantified by Bradford assay (Bio-Rad). Overall, 400–600 μg of protein in 300 μL of Lysis Buffer B (or 250 μg of protein for lipid raft fractions with no extra buffer added) was pre-cleared by rocking over 40 μL of Sepharose 4B beads (Sigma-Aldrich) for 2 h at 4 °C. Supernatants were then rocked over streptavidin-Sepharose beads (ThermoFisher Scientific) overnight at 4 °C. Beads were then washed three times with Lysis Buffer B without protease inhibitor and boiled for 5 min in Laemmli loading buffer supplemented with 2-ME. For precipitations with lipid raft and non-raft fractions, an equal amount of protein was used from each fraction for the assay.

### Glutathione immunoprecipitation

Cells were washed once with PBS/1% BSA and once with PBS, and then incubated in Lysis Buffer B supplemented with 1 mM N-ethylmaleimide for at least 20 min on ice. Protein was quantified by Bradford assay (Bio-Rad). An amount of 300 μg of lysate was brought to 250 μL with lysis buffer. The reduced control was incubated with 50 mM dithiothreitol (+DTT) and rocked at 4 °C for 1 h. The reduced sample was then centrifuged through a Micro Bio-Spin P-6 Gel Column (Bio-Rad). For the IgG control, 5 μg of mouse IgG (Jackson Laboratory) was added to the sample. For all other samples, 2 μg of anti-glutathione antibody (Virogen, Watertown, MA, USA) was added. All samples were rocked overnight at 4 °C. Samples were added to 50 μL of washed Protein G Plus Agarose (ThermoFisher Scientific) and rocked at 4 °C for 1 h. Beads were washed and boiled in Laemmli buffer before being loaded onto a 15% acrylamide gel. Proteins were separated by SDS-PAGE and transferred to a PVDF membrane for immunoblot analysis.

### Metabolic analyses

OCRs and ECARs were measured using the Seahorse XFe 96 Analyzer (Agilent Technologies, Santa Clara, CA, USA) according to the manufacturer’s specifications. Analysis was performed using the Wave Software v2.2.0 or v2.3.0.2 (Agilent Technologies).

### Flow cytometry

For surface staining, cells were washed in PBS and stained with Live/Dead Fixable Blue Dead Cell Stain (ThermoFisher Scientific) for 25 min on ice. Cells were washed and incubated for 25 min on ice with anti-CD25-BV421 (BioLegend, San Diego, CA, USA), anti-CD44-PE (BioLegend), anti CD4-PE-TexasRed (ThermoFisher Scientific), anti-CD8-PerCP-Cy5.5 (BioLegend), anti-TCRβ-PE-Cy7 (BioLegend), and anti-CD45RB-FITC (BioLegend). Cells were washed, fixed in 1% (v/v) methanol-free formaldehyde, and analyzed on an LSRII (BD Biosciences).

For intracellular staining, after staining with Live/Dead Fixable Blue Dead Cell Stain and surface antibodies as described above, cells were washed and fixed with 2% formaldehyde (v/v) for 15 min on ice. Fixed cells were washed and permeabilized with PBS/1% BSA supplemented with 0.03% saponin for 10 min on ice. Cells were washed and incubated with anti-cleaved caspase-3 Alexa 647 (Cell Signaling) for 30 min on ice. Cells were washed, fixed in 1% formaldehyde (v/v), and analyzed on an LSRII (BD Biosciences).

All flow cytometry data were analyzed with FlowJo v10 software (FlowJo, Ashland, OR, USA).

### Cellular and mitochondrial ROS measurement

Cellular ROS was measured using 2′,7′-dichlorodihydrofluorescein diacetate (DCFDA; ThermoFisher Scientific). Overall, 5 × 10^5^ cells were incubated with 1 μM DCFDA in PBS at 37 °C in the dark for 30 min. Cells were washed with cold PBS/1% BSA and analyzed immediately by flow cytometry.

Mitochondrial ROS was quenched using MitoQ^29^. Cell cultures were incubated with MitoQ or a DMSO control for 4 h. Cells were then stained with DCFDA, as described above, for ROS detection.

Mitochondrial ROS was measured using the MitoB probe as previously described^27^. MitoB specifically targets the mitochondria and is converted to MitoP in the presence of ROS. The ratio of MitoP/MitoB was measured using liquid chromatography tandem mass spectrometry.

### Complex I activity and mitochondrial extraction

Cells were washed with PBS/1% BSA and resuspended in STE buffer (250 mM sucrose, 5 mM Tris, 1 mM EGTA, pH 7.4 with HCl). Cells were homogenized and centrifuged at 1000 *g* for 3 min at 4 °C. The supernatant was then centrifuged at 10,000 *g* for 10 min at 4 °C. The supernatant (cytosol) was saved and the pellet (mitochondria) was washed with STE buffer. The mitochondria were then resuspended and assayed for Complex I activity using the Complex I Enzyme Activity Microplate Kit (MitoSciences, Eugene, OR, USA) according to the manufacturer’s specifications. Samples were run in parallel with mouse liver mitochondrial extracts as a positive control. Complex I rates were calculated by dividing Complex I activity by time. Complex I rates were normalized to mouse liver mitochondrial complex I rate.

### Cell death

RICD was induced in day 6 or 7 effector T cells by incubation on plate-bound anti-CD3 (10 μg/mL) for 16–18 h at 37 °C. Cells were removed and stained with Live/Dead Fixable Blue Dead Cell Stain (ThermoFisher Scientific), fixed in 1% formaldehyde (v/v), and analyzed by flow cytometry.

As a positive control for cell death, day 6 effector T cells were incubated with 400 ng/mL FLAG-tagged FasL (Enzo Life Sciences, Farmingdale, NY, USA) and 2 μg/mL anti-FLAG antibody M-2 (Sigma-Aldrich) for 1.5 h at 37 °C. Cells were then stained with Live/Dead Fixable Blue Dead Cell Stain (ThermoFisher Scientific) fixed in 1% formaldehyde (v/v) and analyzed by flow cytometry.

### CD4^+^ T-cell subset differentiation

Purified CD4^+^ T cells were activated in complete medium on plate-bound anti-CD3/soluble anti-CD28 for 2 or 3 days in the presence of differentiating cytokines (Th1: 4 ng/mL IL-12 (PeproTech, Rocky Hill, NJ, USA) plus 10 μg/mL anti-IL-4 (BioLegend); Th2: 10 ng/mL IL-4 (PeproTech) plus 10 μg/mL anti-IFN-γ (BioLegend); Treg: 2 ng/mL TGF-β (PeproTech) plus 100 U/mL IL-2). After differentiation, cultures were propagated for 2 or 3 days in complete medium containing 50 U/mL IL-2 for Th1 and Th2 cells, and 100 U/mL IL-2 for Treg.

### Lipid raft purification

Lipid rafts were separated as previously described^35^. Briefly, cells were lysed on ice for 25 min in TNE buffer (5 mM iodoacetic acid (ThermoFisher Scientific), 150 mM NaCl, 10 mM Tris-HCl pH 7.4, 15 mM EDTA, Complete Protease Inhibitor) supplemented with 100 mM Na_2_CO_3_ and 0.5% Triton X-100. Lysates were sonicated and added to 60% Opti-Prep sucrose substitute (Sigma-Aldrich) to make a final concentration of 40% Opti-Prep. Lysates were placed in an ultracentrifuge tube and layered over with 30 and 5% solutions of Opti-Prep diluted with TNE buffer. Samples were centrifuged for 18 h at 200,000*g* at 4 °C. Eleven 1 mL fractions were taken sequentially from each sample. An equal volume of each fraction was used for immunoblot analysis.

### Influenza infection of mice

Mouse-adapted influenza virus strain A/Puerto Rico/8/1934 H1N1 (PR8) virus (Charles River Laboratories, Wilmington, MA, USA) was used to infect mice. Mice were briefly anesthetized using 2.3% isoflurane in oxygen and infected intranasally with a sublethal dose of PR8 (0.2 LD50) in 0.05 ml of PBS. Control mice received 0.05 ml PBS without virus. Mice were monitored daily until harvest on day 6, at which time the mediastinal lymph node was harvested from the influenza-infected mice, and axillary, brachial, and inguinal lymph nodes were extracted from the PBS control mice. Lymphocytes were collected and stained for analysis by flow cytometry.

### Statistical analysis

Statistical analyses were performed using the graphing software Prism v7 (GraphPad Software, La Jolla, CA, USA). The statistical test used for each experiment is indicated in the figure legends. The following statistical tests were used: paired and unpaired *t*-test when comparing two conditions (e.g., IL-2 compared to IL-15), one-way ANOVA with Tukey test, or Dunnett test (when comparing to one control) for correction for multiple comparisons when comparing multiple conditions for a single variable (e.g., dose titration of 2-DG), two-way ANOVA with Sidak test, or Tukey test for correction for multiple comparisons when comparing multiple variables across multiple conditions (e.g., IL-2 with and without anti-CD3 compared to IL-15 with and without anti-CD3). All data met the assumptions of the statistical tests used and variation between the compared groups was similar.
